The article "A Neural Recording and Stimulation Chip with Artifact Suppression for Biomedical Devices" was published in 2021. Journal: J Healthc Eng.

# A Neural Recording and Stimulation Chip with Artifact Suppression for Biomedical Devices

**DOI:** 10.1155/2021/4153155

**Published:** 2021-08-27

**Authors:** Xu Liu, Juzhe Li, Tao Chen, Wensi Wang, Minkyu Je

**Affiliations:** ^1^College of Microelectronics, Beijing University of Technology, Ping Le Yuan 100# Chao Yang District, Beijing, China; ^2^Advanced Photonics Institute, Beijing University of Technology, Ping Le Yuan 100# Chao Yang District, Beijing, China; ^3^Engineering Research Center of Intelligent Perception and Autonomous Control (Ministry of Education), Beijing University of Technology, Ping Le Yuan 100# Chao Yang District, Beijing, China; ^4^Korea Advanced Institute of Science and Technology, 291 Daehak-ro Yuseong-Gu, Daejeon, Republic of Korea

## Abstract

This paper presents chip implementation of the integrated neural recording and stimulation system with stimulation-induced artifact suppression. The implemented chip consists of low-power neural recording circuits, stimulation circuits, and action potential detection circuits. These circuits constitute a closed-loop simultaneous neural recording and stimulation system for biomedical devices, and a proposed artifact suppression technique is used in the system. Moreover, this paper also presents the measurement and experiment results of the implemented 4-to-4 channel neural recording and stimulation chip with 0.18 *µ*m CMOS technology. The function and efficacy of simultaneous neural recording and stimulation is validated in both *in vivo* and animal experiments.

## 1. Introduction

The neural prosthesis system includes a neural/muscular stimulator and neural recording circuit. These stimulators and recorders of the system have been widely used in many medical fields for decades, such as cochlear/retinal prosthesis, cell activation, and cardiac pacemaker [1–5]. Functionally, neural stimulation is used to activate the prosthesis and wake up the sensory function [6], while neural recording can sense nerve signals or complete the evaluation of stimulation effect [7–9]. Combining neural stimulator and neural recorder, the closed-loop controlled simultaneous neural recording and stimulation system is formed to recover the basic functions of the injured individuals [10–16], such as the system for epileptic seizure detection and suppression [17, 18].

As shown in Figure 1, in the closed-loop neural recording and stimulation system for epileptic seizure detection and suppression, neural recording is used to detect the epileptic signals in brain, and electrical stimulation is used to suppress epileptic seizures. However, the electrical stimulation pulse will cause artifacts and prevent the recording amplifier from normal operation, so the closed-loop system cannot make timely and correct sense-and-trigger response. The problem of stimulation artifact also affects the function of the system in other biomedical devices for brain stimulation and recording [20–22].

### 1.1. Stimulation-Induced Artifact in the Closed-Loop System

To realize multiple functions in biomedical equipment, the neural/muscular recording and stimulation system generally includes multiple recording and stimulation channels, with recording circuits, data processing circuits, stimulation circuits, and electrodes. A bipolar stimulation system is shown in Figure 2(a), which includes a recording circuit with an electrode and a stimulator with one working electrode and one reference electrode. The stimulator with the working electrode provides bidirectional and well-matched stimulation current. During the stimulation, biphasic current flows through the tissue between two electrodes. Therefore, the voltage variation emerges at the stimulation site near the working electrode due to its resistive and capacitive feature. The amplitude of this voltage variation usually ranges from a few hundred millivolts to a few volts, which is mainly determined by the current level and the electrode impedance [23–26]. Then, the voltage waveform generated at the stimulation site has transmitted to the neural recording front end (RFE) through tissue, and it saturates the high-gain recording amplifier. The output signal from the saturated amplifier is called stimulation-induced artefact. The amplifier usually takes a long time to recover from this undesired saturation [23, 24].

Figure 2(b) shows the output voltage waveform of the recording front end, which includes an artifact spike, an artifact tail, and an action potential (AP). This AP has been recorded after the unexpected artifact spike. When the artifact happens, the RFE generally needs 2–10 ms to fully recover and be ready to record the next action potential [27]. Thus, neural recording cannot work normally within this duration, and the next action potential can only be observed after the recording amplifier is fully recovered. Such an artifact problem can be found in most simultaneous recording and stimulation systems [14, 15, 19, 28–30].

### 1.2. Stimulation Artifact Suppression

Several artifact suppression techniques have been reported previously. In the blanking technique [15, 31–34], the RFE is switched off during the stimulation period and turned on during the neural recording. However, the neural signals during the “blanking” period cannot be recorded. In the signal postprocessing technique [35–39], neural signal can be recovered by subtracting the artifact template from the recorded signal. The advantage of the digital processing method is that no neural signal is missed during neural recording. But it is computationally intensive and requests RFE to have a very large dynamic range (several volts) to record artifact signal. In order to obtain a large input dynamic range to record the artifact signal, a track-and-zoom ADC is proposed in [40]. The dynamic input range of RFE is exponentially expanded with the recording signal, which prevents the saturation of neural recording. Another method is to replace the amplifier with a voltage-controlled oscillator (VCO) [41]. This method eliminates the problem of artifact-induced saturation of the amplifier. But the VCO needs further noise optimization to improve the signal-to-noise ratio of neural recording.

Another technique reported is localized stimulation [42, 43]. In this method, the biphasic current can flow through the tissue and return to a local ground. This reduces the artifact amplitude and allows the amplifier to quickly recover to the normal recording state, but the artifact is still not well suppressed. An improved method is dual electrode in-phase stimulation, which carries out differential acquisition at the recording amplifiers [44]. This method has good artifacts suppression effect, but it requires strict impedance matching among the recording electrodes. It is desired to design an extra accurate impedance matching network.

In this paper, we present our implemented closed-loop neural recording and stimulation chip with an artifact cancellation technique. Using the referenced and tuned push-pull stimulation (RTPPS) scheme with a tripolar electrode, the problem of artifact can be solved. A tripolar stimulation configuration with two working electrodes and one reference electrode are used in our method. The stimulation currents delivered by two working electrodes are complementary to each other. By doing so, the impact of large stimulation voltage fluctuation propagated to the recording site can be significantly reduced. The proposed concept is demonstrated with a prototype system including four recording channels and four stimulation channels, in both in vitro and in vivo experiments.

The rest of the paper is organized as follows.  Section 2 explains the proposed stimulation artifact suppression technique and describes the implementation of the prototype recording and stimulation system.  Section 3 presents the bench-top measurement results, as well as the in vitro and in vivo experiment results. Conclusion is given in Section 4.

## 2. Implemented Closed-Loop Neural Prosthesis System with Artifact Cancellation

### 2.1. 4-Channel Neural Recording and Stimulation Chip Implementation

A 4-channel neural recording and stimulation system is designed and presented in this work.  Figure 3 shows the system block diagram. The system consists of four-channel RFEs, four action potential detectors (APD), a global digital (DIG) control block, power down (PD) control, bandgap reference block (BGB) for biasing circuit, and four high-voltage artifact-suppressed stimulators (HVAS). The system can be configured either for multichannel neural recording applications using RFE channels or multichannel neural/muscular stimulation using HVAS channels. With both RFE and HVAS channels active, the system can be configured in four modes: recording (REC), stimulation (STIM), closed-loop recording-stimulation (REC-STIM), and stimulation-recording (STIM-REC). In the REC-STIM mode, the system performs neural signal recording, action potential detection, and action-potential-triggered stimulation. In STIM-REC mode, the stimulator generates stimulation pulses for the specific muscles or neurons, while the RFE is used to monitor stimulation invoked neural signals. In all stimulation-related modes, passive charge balancing (PCB) circuit is used to remove the residual charge after each stimulation pulse to prevent tissue damage. As shown in Figure 3, the PCB circuit is a passive path between the stimulating electrodes and the ground, controlled by CMOS switches. The PCB is only activated at the end of each stimulation pulse.

An artifact cancellation scheme is used in this system design. The so-called RTPPS scheme mentioned in Section 1 aims to cancel the artifact at the stimulation site so that the artifact will not affect the recording site. In conventional bipolar stimulation configuration, the biphasic current (cathodic-then-anodic) flows from a working electrode to a reference electrode. As a result, the stimulation current causes a voltage change at the interface of the working electrodes. This voltage signal is coupled to the input of RFE through tissue and causes artifact. In our implemented stimulator [45], two working electrodes (WE) and one reference electrode (RE) are used to form a tripolar electrode. In this case, the second working electrode counteracts the stimulation from the first working electrode and thus cancels the coupling from the stimulation site to the input of the recording front end. The stimulation currents for the two electrodes are generated by two current generators, namely, the stimulation current generator (SCG) and the countercurrent generator (CCG). By using such stimulation scheme, this system eliminates the voltage fluctuation on the stimulation site and hence reduces the stimulation induced artifact.

### 2.2. High-Voltage Artifact-Suppressed Stimulator

Figure 4 shows the circuit schematic of one stimulator channel, which includes two 10-bit current steering digital-to-analog converters (DACs) and two high-voltage current drivers (HVCD). SCG and CCG have a similar structure and are composed of one DAC and one HVCD. The SCG and CCG produce the same biphasic currents in amplitude to the stimulation target through the electrodes with identical impedance, but with inversed phase. The stimulation pulse width is determined by the timing control of the signals cathodic and anodic in high-voltage current drivers. In the neural stimulator based on constant current stimulation (CCS), the voltage on the electrode depends on the characteristic impedance of the electrode-tissue interface. For larger impedance, HVCD is required. HVCD contains current mirrors with a ratio of 10 to amplify the output current from DAC. The MOS switches connected to the transistors gates are used to activate or deactivate the current generator. To reduce the chip power consumption, the DAC is powered by a 1.8 V supply, and the HVCD is powered by 24 V. The output voltage compliance is therefore large to deliver sufficient stimulation current. The reference voltage is set to a half VDD_h. The current amplitudes of both SCG and CCG are set by DACs and controlled by digital blocks. Besides, the amplitudes of the currents from CCG and SCG are made tunable to compensate for any mismatch between the two electrode interfaces.

### 2.3. Recording Front End and Action Potential Detector

The neural amplifier is one of the most important parts in the neural prosthesis system. As shown in Figure 5(a), the neural recording front end consists of a neural amplifier, a band pass filter (BPF), and a buffer. The capacitor feedback topology with pseudoresistance is selected to achieve low power consumption and low noise. Since the low-pass cut-off frequency of the recording system is determined by the BPF, the bandwidth of the RFE is set to be slightly larger than the nerve signal bandwidth. The gain of the amplifier can be adjusted by the ratio of input capacitance to feedback capacitance. RFE has a programmable gain of 54/60 dB. The high- and low-pass cut-off frequencies can be programmed for different recording modes (spikes only, LPF only, or both). The details of the amplifier design in RFE are described in [46, 47].

The APD is a simple threshold detector, as shown in Figure 5(b). It contains four comparators and two flip-flops (FF). The APD detects both positive and negative spikes, depending on which comes first. The upper 2 comparators and FF are to detect positive spikes. The threshold voltage levels can be tuned by Vtp_H and Vtp_L, and the output trigger signal is asserted when the amplitude of the spike exceeds Vtp_H and becomes nil when the amplitude of the spike drops below Vtp_L as shown in Figure 5(c). This hysteresis window (between Vtp_H and Vtp_L) provides some noise immunity to the detector. Similarly, the lower two comparators and FF are used to detect negative spikes. The hysteresis window can be tuned by Vtn_L and Vtn_H. The trigger signal generated from APD is sent to the digital control block of the system which controls the stimulator. With these two triggering signals from positive and negative threshold detectors, simple spike pattern recognition such as distinguishing biphasic spikes from electrical glitches is enabled.

### 2.4. Digital Control Block

The main functions of the digital control block are to set stimulation parameters and control the stimulation. The digital block has a default command which determines the stimulation parameters such as amplitude and duration. These parameters can also be programmed by an external FPGA through a serial command. The command format, control timing, and function flow of the digital block are shown in Figure 6(a).

Stimulation parameters are decoded from the command frame and stored in global digital control registers. The cathodic and anodic stimulation pulse width (*T*1 and *T*2) use 8-bit control, respectively, and the interphasic delay (Tint) between the two stimulation phases is in 10-bit control. The stimulation current amplitude (VGCM1/VGCM2) control is also in 10-bit. In a typical scenario, several command frames are sent first to configure stimulation parameters. When a spike signal is detected by APD, the embedded finite state machine (FSM) generates control signals such as bs/c < 0 : 4>, Iin_s/c < 0 : 4>, cathodic, anodic, and idle to deliver a predefined biphasic stimulus. After each stimulation pulse, the external switches connect electrodes WE1, WE2, and RE during the idle phase for passive charge balancing (PCB), as shown in Figure 6(b). The interphasic delay between cathodic and anodic phases can be programmed in the range from 0 *μ*s to 255 *μ*s. The detailed stimulation control timing and output waveforms are shown in Figure 6(c). For arbitrary stimulation waveform generation, the pulse width of cathodic and anodic stimulation is divided into 16 steps, respectively, as shown in Figure 6(d). As a result, the current amplitude (D1′–D16′, D1–D16) of each step can be set by sending different commands to the DAC registers.

## 3. Measurement Results

### 3.1. Bench-Top Measurement Results

The 4-to-4-channel closed-loop neural recording and stimulation system is implemented in 0.18-*μ*m high-voltage CMOS technology with LDMOS option. The chip microphotograph is shown in Figure 7. The total chip area is 2 mm by 2 mm.  Figure 8(a) shows the measured output waveforms of two independent HVAS channels of the system. In each channel, the cathodic and anodic current amplitudes are set by two independent 10-bit DACs. It can generate arbitrary stimulation current waveforms including exponential, triangular, ramp, and constant waveforms, respectively, depending on the application requirement. Pulse durations *T*1 and *T*2 are also adjustable in the range from 16 *μ*s to 4 ms.

Figure 8(b) demonstrates test results of the chip configured in the REC-STIM mode. In this configuration, the recording electrodes of RFE and the stimulation electrodes of HVAS are electrically isolated. An ECG signal generated from a function generator is used as a dummy neural action potential signal to the input of one RFE channel. The amplitude of ECG pulse is set as 800 *μ*V peak-to-peak with a frequency of 100 Hz. The gain of RFE is set as 60 dB (1000 V/V). The band-pass filter of RFE is turned off. As shown in Figure 8(c), the APD detects the output of RFE and generates the trigger signal for HVAS. Biphasic stimulation pulses are generated by HVAS and delivered to the electrode nodes, namely, WE1, WE2, and RE. The current waveform is configured as constant current of 600 *μ*A with a pulse duration of 320 *μ*s. The reference voltage on RE is set at 12 (V). A dummy load (a 10 kΩ resistor and a 100 nF capacitor in series) is used between each stimulation output and the reference voltage source.

To demonstrate the proposed artifact-suppression technique, an experiment is done with recording and stimulation electrodes in phosphate-buffered saline (PBS) as shown in Figure 8(c). In the REC-STIM mode, one recording channel is used to record the ECG signal when the ECG spike is detected the stimulator is triggered, delivering the stimulation current to the PBS solution. It is observed that when CCG is disabled, the stimulation artifact saturates the output of the recording amplifier, as shown in Figure 8(d), which needs a long period of time to recover to the normal state before it can perform recording again. However, with CCG enabled in Figure 8(e), an intact ECG signal is recorded during the stimulation period and the saturation is not observed at the output of the recording amplifier.

### 3.2. Animal Experiment

Two in vivo experiments on the rat are carried out using the implemented neural recording and stimulation system. The first experiment is to demonstrate that the artifact generated from muscle stimulation can be suppressed at the input of the recording channel by using RTPPS.

The experiment setup for muscle stimulation is shown in Figure 9(a) [48]. The same chip configuration and ground/power arrangement are used as in Figure 8(c). The recording needle electrode is inserted into the sciatic nerve on the left side of an anesthetized rat, and two concentric stimulation electrodes are inserted in the tibialis anterior (TIB) muscle of the right leg. Two concentric electrodes are put together and share the same reference voltage to form a tripolar stimulation electrode. The voltage waveforms on recording and stimulation electrodes are probed and observed using an oscilloscope. First of all, a biphasic stimulation pulse (amplitude = 90 *μ*A, pulse width = 320 *μ*s) is delivered to the muscle through WE1 and RE by activating SCG only. Figure 9(b) shows the output waveforms at RFE output. It is observed that the stimulation artifact is coupled to the input of RFE through the tissue and saturates its output. Figure 9(c) shows the RFE output when both SCG and CCG are enabled and tripolar stimulation is performed. The artifact is still observed. This is due to the asymmetry between the two electrode-tissue interfaces of WE1 and WE2. In Figure 9(d), the current amplitude generated from CCG is tuned (to a larger value in this case). To compensate the voltage on the recording site due to electrode asymmetry, the pulse width of CCG is divided into 16 steps and the current is different for each step. In the experiment, we tune the current amplitude of each step one by one by sending different commands to the DAC registers, until the artifact voltage cancellation is observed at the recording site. After the tuning, the stimulation artifact is significantly suppressed. Lastly, for comparison, in Figure 9(e), the reference voltage is disconnected from the tripolar electrode configuration to emulate the conventional push-pull bipolar stimulator [42]. In this case, we find that the artifact is a little smaller than the conventional bipolar stimulator, but still cannot be substantially suppressed due to the asymmetry of two stimulation interfaces. In conventional push-pull stimulators, the current tuning is inapplicable since there is no reference point for tuning. Therefore, the shared reference electrode must be present. In aforementioned experiments, successful muscle recruitment on the right foot of the rat is observed.

Another experiment setup for nerve stimulation and recording is shown Figure 9(f), when the system conducts concurrent neural stimulation and recording on the sciatic nerve of an anesthetized rat. The chips configuration and ground/power arrangement are the same as in Figure 8(c). Two concentric electrodes are tied together to form a tripolar (WE1, WE2, and RE) electrode and attached to the sciatic nerve. Note that these two concentric electrodes, however, may not be positioned well within the nerve cross section. This coarse arrangement leads to a possible asymmetric coupling between stimulation and recording sites, which results in asymmetric voltage waveforms at WE1 and WE2 for artifact suppression in this experiment. Two single-needle electrodes are used for recording. One recording electrode is inserted into the nerve which is about 5 mm away from the stimulation site, while the other one is placed in the animal body as a reference. Firstly, a stimulation pulse train is delivered to the nerve from the stimulator. For each pulse, the amplitude is set to 53 *μ*A and the pulse width is 320 *μ*s for both cathodic and anodic phases, with an interphasic delay of 25 *μ*s. Foot dorsiflexion (FD) is observed, and evoked compound action potential (CAP) is recorded. In Figure 9(g), the two test results with and without RTPPS are superimposed in the same graph. The top trace is the stimulation pulse waveform used in RTPPS mode. Middle trace is the recorded RFE response with RTPPS, and the bottom trace is the recorded REF response without RTPPS. Without RTPPS (CCG disabled), the large artifact is caused by saturation of the amplifier and DC voltage drift is observed at the RFE output. When RTPPS is enabled, the stimulation artifact is substantially suppressed. A series of evoked neural spikes can be clearly seen, and the amplitude of the suppressed artifact is reduced to 80–150 mV peak-to-peak, which is only 10%–20% of the CAP signal recorded. The comparison of the prototype neural recording and stimulation chip to prior works is shown in Table 1. It can be found that we have achieved artifact suppression even with a high-gain recorder and large voltage compliance.

## 4. Conclusions

A neural prosthesis chip with stimulation artifact suppression is presented in this work. The implemented 4-to-4 channel neural recording and stimulation system can be configured in recording, stimulation, recording-to-stimulation, and stimulation-to-recording modes, respectively. The function and efficacy of the proposed system has been demonstrated in both bench-top and in vivo experiments. The results show the stimulation induced artifact can be greatly suppressed during closed-loop neural recording and stimulation.

## Figures and Tables

**Figure 1:** Concept of the system for epileptic seizure detection and suppression.

**Figure 2:** (a) Simplified interface between a bidirectional current stimulator and a signal recorder. (b) The output voltage waveform of the recording front end.

**Figure 3:** System block diagram of 4-channel neural recording/stimulation system.

**Figure 4:** Schematic of high-voltage artifact-suppressed stimulator (in each channel).

**Figure 5:** (a) Neural recording front-end (RFE) circuit. (b) Action potential detector circuit. (c) Signal waveforms for functionality illustration of the circuit.

**Figure 6:** (a) Command frame. (b) State machine for stimulator control. (c) Timing and voltage waveforms of control and output signals. (d) Stimulation pulse width division for arbitrary waveform control.

**Figure 7:** 4-channel recording/stimulation IC microphotograph.

**Figure 8:** (a) Arbitrary stimulation waveforms from two HVAS channels. (b) Test-bench measurement results on one channel: output waveforms of recording circuit, APD, and the HVAS stimulator. (c) In vitro test setup and (d, e) Measurement results with and without RTPPS: the top and middle traces show recording outputs from REF channels 1 and 2, respectively. The bottom two traces are the measured voltages on two working stimulation electrodes.

**Figure 9:** (a) In vivo test setup to observe muscle stimulation artifact suppression (recording in sciatic nerve). (b–e) Top traces are the stimulation pulse waveforms, and the bottom trace is the output from RFE. (f) In vivo test setup to observe neural stimulation artifact suppression and (g) test results including comparison to conventional bipolar stimulation.

**Table 1:** Comparison of stimulators for stimulation and recording.

		Reference [49] (REC and STIM)	Reference [50] (REC and STIM)	Reference [37] (REC and STIM)	Reference [40] (REC and STIM)	Reference [24] (REC and STIM)	This work (REC and STIM)
Process		0.13 *µ*m	65 nm	40/0.18 *µ*m HV	0.13 *µ*m	0.18 *µ*m HV	0.18 *µ*m HV
Artifact suppression		Differential acquisition	Digital adaptive filter	ASAR	Track-and-zoom	Resetting RFE	RTPPS
REC	Supply voltage (V)	1.2	1.2/2.5	0.6/1.8/1.2/±5	0.6/1.2/3.3	1	1
	Gain (dB)	—	20	—	92	90	54/60
	Input noise (*µ*Vrms)	2.6	2.9	2.2	1.6	71 nV/rtHz	4.9
	NEF	3.56	—	—	2.86	7.8	2.2
	Power per channel (*µ*W)	0.73	3.21	8.2	1.7	8	4.54

STIM	Compliance voltage (V)	3.3	±11	±8.5	3.3	3/6/9/12	24
	Pulse amplitude (A)	—	2 m	20 *µ*–5.1 m	3 m	5.04 m	1.2 *µ*–1.4 m
	Pulse duration (s)	—	10 *µ*–2 m	10 *µ*–1.28 m	—	15–500 *µ*	16 *µ*–4 m
	Pulse waveform	8 bits, arbitrary	8 bits, arbitrary	8 bits, arbitrary	8 bits, arbitrary	6 bits, arbitrary	5 bits, arbitrary

## Data Availability

The data used to support the findings of this study are available from the corresponding author upon request.
